The article "C-Reactive Protein and High-Sensitive Cardiac Troponins Correlate with Oxidative Stress in Valvular Heart Disease Patients" was published in 2022. Journal: Oxid Med Cell Longev.

# C-Reactive Protein and High-Sensitive Cardiac Troponins Correlate with Oxidative Stress in Valvular Heart Disease Patients

**DOI:** 10.1155/2022/5029853

**Published:** 2022-04-30

**Authors:** Muhammad Ishtiaq Jan, Riaz Anwar Khan, Fozia, Ijaz Ahmad, Naeem Khan, Komal Urooj, Azhar Ul Haq Ali Shah, Asif Ullah Khan, Tahir Ali, Ayesha Ishtiaq, Muhib Shah, Anwar Ullah, Iram Murtaza, Riaz Ullah, Amal Alotaibi, H. C. Ananda Murthy

**Affiliations:** ^1^Department of Chemistry, Kohat University of Science & Technology (KUST), Kohat, Pakistan; ^2^Department of Cardiovascular Surgery, Lady Reading Hospital Peshawar, Pakistan; ^3^Biochemistry Department, Khyber Medical University Institute of Medical Sciences, Kohat, Pakistan; ^4^Department of Biochemistry Abdul Wali Khan University Mardan (AWKUM), Mardan, Pakistan; ^5^Signal Transduction Lab, Department of Bio-Chemistry, Faculty of Biological Sciences, Quaid-i-Azam University Islamabad, Islamabad, Pakistan; ^6^Department of Biochemistry, Bahauddin Zakariya University, Multan, Pakistan; ^7^Institute of Paramedical Sciences, Khyber Medical University, Peshawar, Pakistan; ^8^Department of Pharmacognosy (MAPPRC), College of Pharmacy, King Saud University, Riyadh, Saudi Arabia; ^9^Department of Basic Science, College of Medicine, Princess Nourah bint Abdulrahman University, P.O. Box 84428, Riyadh 11671, Saudi Arabia; ^10^Department of Applied Chemistry, School of Applied Natural Science, Adama Science and Technology University, P.O. Box, 1888 Adama, Ethiopia

## Abstract

**Background:**

Valvular heart disease (VHD) is a major contributor to loss of physical function and longevity. Oxidative stress is one of the key causative factors involved in heart disease including VHD. Here, we aimed to illuminate the role and relation of oxidative stress to the VHD risk markers in the human population.

**Materials and Methods:**

150 VHD patients and 103 healthy individuals as control were selected for the study and were divided into three groups: the aortic valve, mitral valve, and combined disease based on valvular calcification.

**Results:**

Our results demonstrated enhanced oxidative stress in the VHD condition, as we found elevated levels of reactive oxygen species (ROS) at the serum, supported by an increased level of thiobarbituric acid reactive substances (TBARs) in the cardiac valvular tissues of the VHD patients. In contrast, we experienced declined antioxidants including Super Oxide Dismutase (SOD), catalase (CAT), and peroxidase (POD) activities. Concurrently, increasing levels of C-reactive protein (CRP), high-sensitivity cardiac troponin I (hs-cTnI), and high-sensitivity cardiac troponin T (hs-cTnT) were detected in the aortic, mitral, and combined disease condition, suggesting a key association of oxidative stress to VHD conditions. Furthermore, regression analysis validated a key association between the impairment of the redox system (ROS and antioxidant enzyme activities) and VHD condition.

**Conclusion:**

Taken together, dysregulated oxidative stress contributes to the progression of VHD via positively correlating with CRP, hs-TnI, and hs-TnT level.

## 1. Introduction

VHD is the leading cause of death for men and women in developing countries, including Pakistan. Aortic valve dysfunction leads to left ventricular overload. However, the ventricle creates a hypertrophic response to counteract the hemodynamic pressure, leading to an increase in myocyte size, mass, and wall thickness [1]. In addition, the left atrial enlargement is also observed in patients with aortic stenosis [2]. Left atrial enlargement reflects the left atrium's pressure overload, which is also an established marker of chronically increased hemodynamic burden [3]. Left atrial pressure or volume overload also occurs due to mitral valve disease. Left atrial remodeling and enlargement occur due to persistently maintained pressure overload in the left atrium [4].

In addition, a variety of natriuretic peptides, including NT-proB-type natriuretic peptide (NT-ProBNP), atrial natriuretic peptide (ANP), and B-type natriuretic peptide (BNP), are secreted during hypertrophy of the left ventricle and left atrial dilation, which can be used as powerful hypertrophic markers of the heart in the blood [5, 6]. Additionally, CRP is an inflammatory marker of the plasma protein responsive component. The elevated level of CRP is also associated with left ventricular hypertrophy [7] and left atrial enlargement [8]. Furthermore, hs-cTnI and hs-cTnT are reliable indicators of subclinical and ongoing myocardial damage. These biomarkers are associated with the progression of hypertrophic cardiomyopathy leading heart failure [9].

The calculation damages the valve leaflets, and the increase in oxidative stress is reported to play a significant role in the breakdown of smooth muscle tissue into an osteoblast-like phenotype [10]. However, hydrogen peroxide acts as a proinflammatory second messenger and involves in the osteogenic mineralization of smooth muscle cells [11]. In addition, ROS is a key player in inflammatory diseases [12]. However, previous literature study showed that in addition, ROS is a key player in inflammatory diseases [13]. Initially, ROS is generated as a response to any stimuli or defense mechanism that leads to enhanced inflammation in dysregulated conditions, as reported [14] via JNK signaling [15]. It suggests a key link between ROS and inflammation. Furthermore, respiratory bursts made by inflammatory cells during inflammation lead to increased production and accumulation of ROS at the site of damage [16, 17]. The intracellular antioxidant enzymes play a significant role in neutralizing the oxidative stress [18]. The former reports about the increased generation of ROS, and reduced antioxidant potential in different cardiac diseases evoked the current study. Furthermore, in our previous study, we reported a causative relationship of ROS to cardiomyocyte apoptosis [19]. Therefore, in the current study, we aimed to evaluate the oxidative stress in VHD patients and found elevated ROS and biomarkers, CRP, hs-cTnI, and hs-cTnT, while the decline in antioxidant enzyme activities was found in VHD patients suggesting a key role of oxidative stress in the progression of cardiac hypertrophy due to VHD.

## 2. Material and Methods

### 2.1. Study Population

Data and blood samples were collected from patients received between June and December 2019 for valve insertion at the Cardiovascular Department, Lady Reading Hospital, Peshawar, Pakistan. Patients were not included in the study which showed a history of myocardial infarction, complex diabetes, other diseases developed by the coronary artery, and kidney failure. The Institutional Ethics and Clinical Research Committee of Lady Reading Hospital (Peshawar, Pakistan) approved the current study. In this study, informed written consent was given to patients prior to participation. However, in human studies, research was conducted in accordance with the 1975 Helsinki Declaration. A total of 150 patients were selected for severe stenosis, regurgitation, and joint disease status. In addition, patients were divided into three main groups on the basis of complex calculation, aortic valve disease (aortic valve replacement, AVR), mitral valve disease (Mitral valve replacement, MVR), and diseases involving the condition of the aortic and mitral valve (double valve replacement (DVR)). The mean age of the patients was 45.6 ± 12.4 years and 48.3 ± 10.5 years for men and women, respectively. In addition, samples were also collected from 103 average people, including men and women aged 44.3 ± 10.4 and 46.1 ± 11.3. The New York Heart Association (NYHA) classification criteria were used to address the severity of chronic heart failure in aortic and mitral valve patients [20].

### 2.2. Baseline Diagnosis and Severity of Valve Diseases

Initial diagnosis and evaluation were performed with chest X-ray and CT scan. A standard grade five calcification was observed during image interpretation in all patients [21]. Besides, the severity of valve dysfunction was observed through different standard parameters during transthoracic echocardiography [22].

### 2.3. Biochemical Analyses

#### 2.3.1. ROS Assay

Serum ROS levels were measured using a method previously developed by Hayashi et al. [23]. Reagent 1 was prepared by dissolving 10 mg of N, N-diethyl-paraphenylenediamine (DEPPD) in 100 mL of 0.1 M sodium acetate buffer. Reagent 2 was prepared as a stock solution of ferrous sulfate by dissolving 50 mg of ferrous sulfate in 10 mL of acetate buffer. Form the stock, Reagent 2 was prepared by adding 50 *μ*L of solution in 100 mL of acetate buffer. N, N-Diethyl-paraphenylenediamine was used as a chromogenic solution and ferrous sulfate as a transition iron ion. Both the reagents were mixed in a ratio of 1 : 25 and stored in the dark for 20 minutes. Reagent (1680 *μ*L), buffer (1200 *μ*L), and serum sample (60 *μ*L) were taken in a cuvette. Different concentrations of hydrogen peroxide were used to form a standard curve. The reading was observed with a 15-second interval for each sample. Absorbance was measured by using a spectrophotometer at 505 nm in triplicate.

#### 2.3.2. SOD Assay

SOD was measured as described earlier by Beyer and Fridovich [24]. L-Methionine, NBT.2HCl, and Triton X-100 were mixed with phosphate buffer saline. A fixed amount of this solution was then mixed with serum and illuminated with a fluorescent light. After incubation at 37°C, cooled riboflavin was added and placed at 40°C to initiate the reaction. Absorbance was then recorded three times per sample with a spectrophotometer of 560 nm after a 1-minute interval.

#### 2.3.3. CAT Assay

CAT activity was measured using hydrogen peroxide as a substrate described by Aebi et al. [25]. Potassium phosphate buffer, hydrogen peroxide, and serum sample were mixed. Sample absorption was detected at 240 nm three times with a time interval of 30 seconds. The activity of one catalase unit is defined as an absorption change of 0.01 as a unit per minute.

#### 2.3.4. POD

POD activity was measured by preparing the reaction mixture of phosphate buffer, guaiacol, and a serum sample. Hydrogen peroxide is added to the mixture, and the absorption rate is measured at 420 nm after 60 seconds. Absorbance was seen as a minute change in absorption [26].

#### 2.3.5. Ascorbate Peroxidase Assay

Ascorbate peroxidase (APX) testing was performed by mixing samples of serum, potassium phosphate buffer, EDTA, ascorbate, and hydrogen peroxide. Absorption of ascorbate reduction was measured at 290 nm in triplicate [27].

#### 2.3.6. TBARs Assay

TBARs assay was performed as described by Buege and Aust in [28]. A serum sample was mixed with FeSO_4_, Tris-HCl, and ascorbic acid. The reaction mixture was reconstituted after the administration of trichloroacetic acid and thiobarbituric acid. The reaction mixture was centrifuged, and the supernatant absorption was measured at 532 nm.

#### 2.3.7. Measurements of CRP and High-Sensitivity Cardiac Troponin Biomarkers

Serum samples were collected after centrifugation of plasma samples at 15000 rpm for 10 min. CRP levels were measured by a validated Human C-Reactive Protein ELISA Kit (Invitrogen). The samples were processed according to the instructions provided with the kit. In addition, total cholesterol, triglycerides, and high-density lipoprotein cholesterol (HDL-cholesterol) were also measured. Both the biomarkers cTnI and cTnT were processed according to the manufacturers' instructions and reported within 24 hours after the collection of blood samples. Serum hs-cTnI is measured with ARCHITECT STAT High Sensitive Troponin-I assay (Abbott Diagnostics). Serum hs-cTnT was measured with Elecsys Troponin T-High Sensitive immunoassay (Roche Diagnostics Ltd., Rotkreuz, Switzerland).

#### 2.3.8. Statistical Analysis

The data was displayed as a standard ± standard definition (SEM). The SPSS 21 service (IBM Corp., Armonk, NY, USA) was used to analyze statistics between different groups. *P* < 0.05 was considered significant.

## 3. Results

### 3.1. Baseline Characteristics

The prevalence of VHD was higher in male than female patients in the age-matched individuals (patient/control). However, in total cases, the aortic valve disease condition was high in male while mitral valve disease was high in female patients. The combined disease condition of the aortic and mitral valve was high in male as compared with female patients as shown in Figure 1. Here, we employed patients with severe aortic, mitral, and combined disease conditions of both valves due to calcification and were classified into class III (91.%) and class IV (9.9%) according to the New York Heart Association (NYHA) classification criteria given in Figure 2.

### 3.2. Redox System Impairment in the VHD Patients

Due to excessive free radical generation and declined antioxidant defense mechanism, the dysregulated redox system could contribute to different diseases, including cardiovascular abnormalities. Herein, we found an increased level of ROS in VHD patients (aortic valve, mitral valve, and both the disease conditions of aortic and mitral valve patients) compared to the normal individuals (Figure 3(a)). However, contrary to oxidative stress, we found decreased activities of the antioxidant's enzymes, including SOD, CAT, POD, and the APX, in the patients with VHD (Figures 3(b)–3(e), respectively). Furthermore, elevated levels of TBARs in the VHD patients validated the oxidative stress relation to VHD concurrently (Figure 3(f)). Notably, our regression analysis further demonstrated a negative correlation of ROS and antioxidant enzyme activities in the VHD conditions as shown in Figure 4. Overall, these data suggest a causative relationship of redox system impairment in VHD conditions.

### 3.3. VHD Patients Displayed Increased Levels of CRP and High-Sensitive Cardiac Troponin

CRP is a well-known inflammatory marker of several cardiovascular diseases, including cardiomyopathy. Herein, we measured CRP levels in the VHD patients and detected elevated CRP levels in all three forms of VHD, including aortic, mitral, and combined aortic and mitral valve disease. Similar to CRP, high-sensitive cardiac troponin is an established heart dysfunction and risk marker. We also measured both hs-cTnI and hs-cTnT level in the VHD patients. Interestingly, these markers significantly increased in both the aortic and mitral valve diseases, indicating a key relation to VDH and suggesting an increased risk of left atrial enlargement and left ventricular hypertrophy due to aortic and mitral valve dysfunction. Concurrently, we found impaired levels of total cholesterol, Tg, and HDL, further validating valvulopathy in our employed subjects (Table 1).

Next, we performed correlation analysis of ROS and VHD risk markers, including CRP, hs-cTnI, and hs-cTnT. Interestingly, we found a significant positive correlation between ROS and these risk factors, demonstrating that oxidative stress is the key factor involved in the VHD and its progression (Figure 5).

## 4. Discussion

In the present study, we demonstrated a causative relationship, between oxidative stress and VHD, by measuring ROS level and antioxidant activities. The increased ROS level was positively correlated with CRP, hs-cTnI, hs-cTnT, and lipid level impairments; however, ROS were negatively correlated with antioxidant enzyme activities in the VHD patients. ROS plays a vital role in cell signaling as a mediator and regulator of vascular function; however, impaired levels of ROS contribute to various cardiac complications. Several signaling modulators related to soft tissue calcification [29], inflammation [30], and matrix remodeling [31] are activated in response to ROS dysregulation. In the early stages of heart valve disease, oxidative stress may contribute to the development of myofibroblast [32]. These activated cells are later divided into cells with similar properties to osteoblast. In vitro research confirms evidence of osteoblast-like phenotype. In addition, an increase in the formation of numbered nodules on vascular muscle was observed with an increase in oxidative stress [29]. Therefore, it can be speculated that oxidative stress may be high in many manifestations leading to changes in features such as osteoblast aortic valve. Similarly, increased levels of ROS have been found in the identified areas of stenotic aortic valves, which play an important role in local inflammatory response [30, 33].

In the present study, we found significantly high levels of ROS in respective groups of aortic, mitral, and combined aortic with mitral valve diseases. The high levels of serum ROS may also be due to severe calcification and inflammation in the aortic and mitral valves. The low antioxidant enzymatic activity of SOD may also contribute to the high activity of oxidative stress in the serum of VHD patients. In addition, antioxidant enzymatic activities of CAT were found low in cardiac valve patients of present study cohorts. Likewise, the low activity levels of SOD were also observed in all the disease groups of VHD patients. The low activity levels of POD enzymatic activities have also been studied in different pathological conditions of cardiovascular diseases [34]. However, in the present study, low levels of POD enzymatic activity were also identified in all appropriate disease groups of VHD patients. Reduced SOD activity levels are either due to low SOD exposure [35] or due to impairment of processes that regulate SOD expression, e.g., peroxisome proliferator-activated receptor gamma [36] or paradoxical reductions in proinflammatory stimuli that occur in late-stage aortic valve stenosis [37]. The low activity of APX is related to the increased risk of cardiovascular diseases [38]. In this study, the low activity of APX was identified in disease groups of VHD patients, which is followed by the previous data. The high levels of ROS result in cardiomyocytes damage and apoptosis due to their direct oxidizing effects on proteins, lipids, and DNA [39–41]. In addition, the increased ROS leads to lipid damage, which is the early indicator of different heart diseases [42]. In the current study, the TBARs activity was found significantly high in all the aortic and mitral valve disease groups. In addition, according to regression analysis, ROS activity showed a negative relationship with antioxidant activities while on the other hand, a positive relationship was found with TBARs which suggests the role of reactive oxygen species in the development of aortic and mitral valve calcification leading to VHD.

The independent association between CRP level and cardiac hypertrophy is consistent with previous results [7]. We have previously published the association between left atrial enlargement and left ventricular hypertrophy with ANP and BNP [5], but herein, the CRP observation is extended to left atrial enlargement and left ventricular hypertrophy due to the aortic and mitral valve dysfunction. However, it is believed that CRP may also be a potent marker for the detection of cardiovascular diseases. The increased level of CRP has been associated with inflammation and endothelial dysfunction [43], which ultimately promotes an increase in cardiac mass. It is speculated that CRP signals cardiac hypertrophy by promoting phosphatidylinositol-3 kinase activity [44], inducible nitric oxide synthase, mitogen-activated protein kinase pathway, and nuclear factor *κ*-B. Both the biomarkers hs-cTnI and hs-cTnT are independently associated with hypertrophic cardiomyopathy; however, hs-cTnI provides robust information about cardiac hypertrophy [45]. In the present findings, the levels of both the hs-cTnI and hs-cTnT were significantly high in all the disease groups of the aortic and mitral valve. The high levels of both the markers are may be due to the left atrial enlargement or left ventricular hypertrophy. In addition, the high levels of both the markers may also be due to combined disease condition of both the left atrial enlargement and left ventricular hypertrophy due to the dysfunction of respective valves. It is therefore observed that the concentration of both the hs-cTnI and hs-cTnT was high in combined disease conditions when compared with a single disease condition. In the present study, there are strong associations of hs-cTnI and hs-cTnT with cardiac hypertrophic [46, 47]. We suggest here, on the basis of previous and present findings, that both hs-cTnI and hs-cTnT can be used as a potent diagnostic biomarker for the assessment of left atrial enlargement and left ventricular hypertrophy. To the best of our knowledge, we have demonstrated the association between hs-cTn with left atrial enlargement and left ventricular hypertrophy due to the dysfunction of aortic and mitral valves.

## 5. Conclusion

Overall, this analysis demonstrated that dysregulated oxidative stress could contribute to valvular heart damage via cellular signaling disruption. Under oxidative stress conditions, the decline of antioxidant enzyme activities exaggerated CRP, hs-cTnI, and hs-cTnT levels, indicating left atrial enlargement followed by left ventricular hypertrophy. Furthermore, impaired levels of VHD risk markers (CRP, hs-cTnI, and hs-cTnT) correlated with ROS, providing relevant prognostic information that may be helpful to refine CVD risk stratification.

## Figures and Tables

**Figure 1:** Prevalence of aortic valve disease in male and female patients. (a) Aortic valve disease is high in male patients. (b) Mitral valve disease is high in female patients. (c) The disease condition of both the aortic and mitral valves is high in male compared with female patients.

**Figure 2:** New York Heart Association classification of patients showing 91.1% patients in class III and 8.9% patients in class IV.

**Figure 3:** ROS and antioxidant activity levels. (a) The level of ROS is significantly high in aortic, mitral, and combined disease condition. (b) The activity of SOD is significantly low in all the three respective disease conditions. (c) The activity of CAT is significantly low in all the disease conditions of aortic, mitral, and combined disease condition of aortic with mitral valves. (d) The activity of POD is significantly low in all the disease groups of aortic and mitral valve. (e) The level of APX is significantly low in all the pathological conditions of aortic and mitral valve. (f) The level of TBARs is significantly high in all the respective disease groups of the aortic and mitral valve.

**Figure 4:** Regression analysis between ROS, antioxidant, and TBARs activity levels: (a) ROS vs. SOD in AVR; (b) ROS vs. SOD in MVR; (c) ROS vs. SOD in DVR; (d) ROS vs. catalase in AVR; (e) ROS vs. catalase in MVR; (f) ROS vs. catalase in DVR; (g) ROS vs. POD in AVR; (h) ROS vs. POD in MVR; (i) ROS vs. POD in DVR; (j) ROS vs. APX in AVR; (k) ROS vs. APX in MVR; (l) ROS vs. APX in DVR; (m) ROS vs. TBARS in AVR; (n) ROS vs. TBARs in MVR; (o) ROS vs. TBARs in DVR. AVR: aortic valve replacement; MVR: mitral valve replacement; DVR: double valve replacement.

**Figure 5:** Regression analysis of ROS with CRP, hs-TnI and hs-TnT: (a) ROS activity vs. CRP in AVR; (b) ROS activity vs. CRP in MVR; (c) ROS activity vs. CRP in DVR; (d) ROS activity vs. hs-TnI in AVR; (e) ROS activity vs. hs-TnI in MVR; (f) ROS activity vs. hs-TnI in DVR; (g) ROS activity vs. hs-TnT in AVR; (h) ROS activity vs. hs-TnT in MVR; (i) ROS activity vs. hs-TnT in DVR. AVR: aortic valve replacement; MVR: mitral valve replacement; DVR: double valve replacement.

**Table 1:** Clinical characteristics of patients vs. controls.

	Aortic valve disease		Mitral valve disease		Aortic+mitral valve disease	
	Patient	Control	Patient	Control	Patient	Control
M/F	21/6	16/5	27/52	21/28	27/17	20/13
Age (years)	49.7 ± 10.1	47.7 ± 9.1	44.2 ± 11.9	43.8 ± 10.2	48.5 ± 12.1	46.3 ± 11.8
hs-cardiac Trop I ng/mL	0.044 ± 0.01	0.029 ± 0.02	0.041 ± 0.01	0.030 ± 0.01	0.051 ± 0.02	0.022 ± 0.01
*P* value	0.001^∗∗^	—	0.00^∗∗^	—	0.00^∗∗^	—
hs-cardiac Trop T ng/mL	0.048 ± 0.02	0.022 ± 0.01	0.051 ± 0.02	0.026 ± 0.01	0.060 ± 0.01	0.048 ± 0.02
*P* value	0.02^∗^	—	0.00^∗∗^	—	0.00^∗∗^	—
CRP mg/L	4.2 ± 0.87	2.9 ± 0.73	4.4 ± 1.17	2.8 ± 0.89	4.9 ± 1.14	3.0 ± 0.63
*P* value	0.03^∗^	—	0.02^∗^	—	0.00^∗∗^	—
Total cholesterol (mmol/L)	5.13 ± 0.09	5.32 ± 0.07	5.29 ± 0.08	5.11 ± 0.07	5.33 ± 0.09	5.23 ± 0.08
*P* value	NS	—	NS	—	NS	—
Triglyceride (mmol/L)	1.53 ± 0.07	1.49 ± 0.06	1.61 ± 0.08	1.65 ± 0.07	1.71 ± 0.06	1.81 ± 0.09
*P* value	NS	—	NS	—	NS	—
HDL cholesterol	1.45 ± 0.09	1.57 ± 0.07	1.67 ± 0.08	1.57 ± 0.06	1.78 ± 0.08	1.81 ± 0.07
*P* value	NS		NS		NS	

Values are given as mean ± SEM; ^∗∗^*P* < 0.01 and ^∗^*P* < 0.05.

## Data Availability

All the available data are incorporated in the MS.
